# Akt2 Regulates the Differentiation and Function of NKT17 Cells via FoxO-1-ICOS Axis

This article has been retracted.

**DOI:** 10.3389/fimmu.2018.01940

**Published:** 2018-09-12

**Authors:** LinLin Niu, Xingtian Xuan, Jinzhi Wang, Liling Li, Di Yang, Yukai Jing, Lisa S. Westerberg, Chaohong Liu

**Affiliations:** ^1^Chongqing Key Laboratory of Child Infection and Immunity, Chongqing, China; ^2^Department of Pediatric Research Institute, Children's Hospital of Chongqing Medical University, Chongqing, China; ^3^Ministry of Education Key Laboratory of Child Development and Disorders, Chongqing, China; ^4^Department of Pathogen Biology, School of Basic Medicine, Huazhong University of Science and Technology, Wuhan, China; ^5^Department of Microbiology Tumor and Cell Biology, Karolinska Institutet, Stockholm, Sweden

**Keywords:** Akt2, iNKT, ICOS, NKT17, FoxO-1

## Abstract

As a critical linker between mTORC1 and mTORC2, Akt is important for the cell metabolism. The role of Akt in the function and development of B and T cells is well characterized, however, the role of Akt for development and function of iNKT cells is unknown. iNKT cells bridge the adaptive and innate immunity, and in this study, we found that the differentiation of NKT17 cells and IL17 production of NKT17 cells were disrupted in Akt2 KO mice. ICOS has been demonstrated to be critical for the differentiation of NKT17 cells and we found that ICOS mRNA and protein expression was reduced in Akt2 KO iNKT cells. As a consequence, phosphorylation of FoxO-1 was downregulated in Akt2 KO thymocytes but the sequestration of FoxO-1 in the nucleus of Akt2 KO iNKT cells was increased. The negative feedback loop between ICOS and FoxO-1 has been demonstrated in CD4^+^T follicular helper cells. Therefore our study has revealed a new intracellular mechanism in which Akt2 regulates ICOS expression via FoxO-1 and this signaling axis regulates the differentiation and function of NKT17 cells. This study provides a new linker between cell metabolism and function of iNKT cells.

## Introduction

The invariant NKT(iNKT) cells have a critical role to bridge the innate and adaptive immunity. They are generated in thymus and unique αβ T cells characterized by the expression of a semi-invariant TCRα and TCRβ chain with limited repertoire (1, 2) that binds to endogenous, microbial, and synthetic lipid ligands presented by CD1d. Traditionally the development of iNKT cells can be divided into 4 different stages from stage 0 to stage 3 according to the surface molecules of CD24, CD44 and NK1.1. These include immature stage 0 (CD24^+^CD44^−^NK1.1^−^), to transitional stage 1(CD24^−^ CD44^−^NK1.1^−^), to stage 2 (CD24^−^CD44^+^NK1.1^−^), and finally to mature stage 3 (CD24^−^CD44^+^NK1.1^+^) (3). Many transcriptional factors have been identified to have an indispensible role for iNKT cell development. PLZF, the most notable example, is crucial for the early development and functional differentiation of iNKT cells (4, 5). iNKT cells can be categorized into three lineages according to the expression of the transcriptional factors T-bet, GATA3 and RORγt to define NKT1, NKT2, and NKT17 cells respectively (6, 7). Although many regulators of iNKT cell development has been identified, the relationship between developmental maturation and lineage diversification still remains elusive.

The Akt family of proteins consists of three isoforms named Akt1, Akt2, and Akt3 (8), and they share similar structure and function (9). They promote cellular metabolism and positively regulate cell proliferation and survival via activation of downstream signaling molecules (10). The activation of Akt requires the activation of the upstream signaling molecule PI3K (11). Akt has been shown to be indispensible for the development and differentiation of T cells and B cells (12–14). Thymocyte progenitors lacking Akt1 and Akt2 fail to effectively transit from DN3 stage to the double positive stage (12, 13). Although the generation of downstream precursors from Akt1/2 deficient pro-B cells is not affected, the selection of MZ B cells and the survival of mature B cells are impaired (14). However the role of Akt2 in the development of iNKT cells has not been investigated so far.

One of the major downstream pathways of PI3K signaling is the Akt-mediated inactivation of transcriptional factors FoxO-1 (14). Akt mediated phosphorylation of FoxO-1 causes the exit of FoxO-1 from nucleus to the cytoplasm where it undergoes ubiquitin mediated degradation (15). FoxO-1 is critical for the expression of cyclin dependent kinase inhibitors and proapoptotic genes (16, 17). FoxO-1 has been shown to positively regulate growth factor receptors including the expression of IL7Ra (18). In turn, signals through PI3K induce FoxO-1 inactivation, which generates a negative feedback loop (17, 19). FoxO-1 has been shown to regulate the ICOS expression by binding to the consensus binding site of T cell co-stimulator (ICOS) and remain bound after activation for 48 h (20). Inducible ICOS is a co-receptor similar to CD28 and induced in activated T cells, and highly expressed in T follicular helper (Tfh) cells. ICOS signaling is important for the development of GC B cells, T cell dependent B cell help and antibody class switching (21). Signal transduction through ICOS results in the activation of PI3K (22). Whether the axis of ICOS-Akt-FoxO-1 has any role in the development and function of iNKT cells remains to be determined.

In our study, we used Akt2 KO mice as a model to study the effect of Akt2 deficiency on the development and function of iNKT cells. We found that the homeostasis of iNKT cells and the differentiation of NKT17 cells was impaired and associated with reduced IL-17 production. Furthermore, we found that the reduction of iNKT cells was due to increased apoptosis and reduced proliferation with increased Bcl2 expression. We define the mechanism by showing that the ICOS-Akt-FoxO-1 axis was impaired in Akt2 KO iNKT cells and this leads to a reduction in NKT17 cells.

## Materials and methods

### Mice

Akt2 KO and Icos KO mice were purchased from Jaxson Laboratory. All mice were kept in the specific pathogen—free conditions in the animal center of Children's Hospital of Chongqing Medical University. The 4- to 8- week old Akt2 KO or Icos KO mice and the wild type (WT) littermates were used for the studies. All animal experiments were performed according to protocols approved by the Institutional Animal Care and Usage Committee of Children's Hospital of Chongqing Medical University.

### Flow cytometry

Thymocytes and splenocytes were made according to the published protocols (23). Cells were stained for surface markers with the following monoclonal antibodies: phycoerythrin (PE)-conjugated mouse CD1d tetramers loaded with PBS-57 were provided by the NIH Tetramer Facility. FITC-anti-mouse CD44 (IM7), APC-anti-NK1.1 (PK136), PE-Cy7-anti-CD24 (M1/69), APC-Cy7-anti-TCR-β (H57-597), PB-anti-CD4 (RM4-5), BV510-anti-CD8 (53-6.7), FITC-anti-Annexin V, Percp-anti-CD45.2 (104), APC-anti-CD45.1 (A20), PB-anti-CD45.1 (A20), PB-anti-CD45.2 (104), PE-Cy7-anti-CD45.2 (104), and PE-Cy7-anti-CD45.2 (A20) antibodies were purchased from Biolegend. Percp-anti-7AAD antibody was purchased from BBIlife sciences. Cell surface staining was made in 2% (vol/vol) FBS-PBS, All the cells were incubated on room temperature for 30 min.

### Phospho flow

Thymocytes were incubated with Percp-anti-7AAD (BBIlife sciences), PE-Cy7-anti-CD44 (IM7; Biolegend), APC-Cy7-anti-TCR-β (H57-597; Biolegend), PB-anti-CD4 (RM4-5; Biolegend), and BV510-anti-CD8 (53-6.7; Biolegend) antibodies at 4°C for 30 min and pulsed at 37°C water bath for 5, 15, and 30 min with PMA (50 ng/ml) and Ionomycin (500 ng/ml). The cells were fixed, permeabilized, and stained with phosphorylated FoxO-1 (pFoxO-1, S256; Cell Signaling technology) for 1 h, and further stained with an AF488-Goat anti-rabbit (Life technology) secondary antibody for 30 min.

In order to analyze the phosphorylated level of STAT3, thymocytes were stimulated with PMA and Ionomycin or α-GalCer. For PMA and Ionomycin stimulation, thymocytes were incubated with PMA (50 ng/ml) and Ionomycin (500 ng/ml) in 37°C water bath for 5, 15, and 30 min. For α-GalCer stimulation, thymocytes (2 × 10^6^) were seeded in a 24-well plate in 1640+10% FBS with the addition of α-GalCer (125 ng/ml) for 72 h. PE-anti-STAT3 phospho (pSTAT3, Tyr705; Biolegend) were analyzed. The cells were fixed, permeabilized, and stained with PE-anti-STAT3 phospho (pSTAT3, Tyr705; Biolegend) for 1 h. All flow cytometry data were collected using a FACS Canto (BD Biosciences) and analyzed with FlowJo software. Mean fluorescent intensity is indicated.

### Enrichment of iNKT cells

For *ex vivo* stimulation, iNKT cells need to be enriched from thymocytes and splenocytes by depleting CD8α^+^ cells. Briefly, the total thymocytes in 200 μL of Hank's Balanced Salt (HBSS) were incubated with CD8α (Ly-2) MicroBeads (Miltenyi Biltec) on ice for 15 min, and iNKT cells were enriched using LS columns (Miltenyi Biltec) according to the manufacturer's protocol. The enriched cells were used for surface staining of PE-anti-ICOS (TE.17G9, eBioscience), PE-anti-IL-23R (12B2B64), and FITC-anti-Annexin V (Biolegend). Intracellular staining for PLZF, RORγt, T-bet, GATA3, Bcl2, Ki-67, and c-Maf was fixed and permeabilized using a Foxp3 Staining Buffer Set (eBiosciense). For α-GalCer stimulation, thymocytes (6 × 10^6^) and splenocytes (6 × 10^6^) were seeded in a 24-well plate in 1640+10% FBS, left unstimulated, or stimulated with α-GalCer (125 ng/ml) for 72 h, with the addition of PMA (50 ng/ml) and ionomycin (500 ng/ml)in the last 5 h. After stimulation, cells were stained with CD1d, TCRβ, CD44, NK1.1, IFN-γ, IL-17a, IL-4, and TNFα.

### qRT-PCR

Total RNA was isolated from the sorted CD4 positive T cells using TRIzol Reagent (BioTeke) and was reversely transcribed using the PrimeScript™ RT Reagent Kit (Perfect Real Time) (TaKaRa). qRT-PCR were performed with the Hamburg (Eppendorf) PCR and CFX96 Real-Time System (Bio-Rad) with the following primer pairs: *icos* (5′-CTCACCAAGACCAAGGGAAG-3′ and 5′-CTTGAAAAGGAGGTGGGTCA-3′), *c- maf* (5′-GAGGAGGTGATCCGACTGAA-3′ and 5′-TCTCCTGCTTGAGGTGGTCT-3′), *thpok* (5′-TCTCCTGCTTGAGGTGGTCT-3′ and 5′-CTCGCTCACAGTCATCCTCA-3′). For the relative mRNA expression level of *akt2* gene, CD4^+^T cells, CD19^+^B cells, iNKT cells and NKT17 cells (stage2 ICOS^+^ iNKT cells) were sorted using a FACSAria™II (BD Biosciences). The primer pairs: *akt2* (5′-CCCTGACCAGACCTTACC-3′ and 5′-TGCCGAGGAGTTTGAGATA-3′). Expressed levels of target mRNAs were normalized with GAPDH and calculated using the 2^−ΔΔCT^ method.

### Immunofluorescence microscopic analysis

For α-GalCer stimulation, the sorted iNKT cells were seeded in a 96-well plate in DMEM (with 10% FBS), left unstimulated, or stimulated with α-GalCer (125 ng/ml) for 72 h. α-GalCer -stimulated iNTK cells were dropped on the poly-L-lysine slides, incubated for 30 min, fixed with 4% paraformaldehyde, and then permeabilized with 0.05% PB buffer. The unstimulated iNKT cells were incubated with a mouse anti-PLZF antibody (4 μg/ml, Santa Cruz Biotechnology) and AF488-Actin (Invitrogen) for 1 h, further stained with a Goat anti-mouse AF546 secondary antibody (1:400) for 30 min, and finally covered with 1.5 μg/ml DAPI (Beyotime). α-GalCer stimulated iNTK cells were incubated with rabbit-anti-FoxO-1 (Cell signaling technology) and AF488-Actin for 1 h, and further stained with a AF546-Goat anti-rabbit secondary antibody (1:400) for 30 min, and finally covered with 1.5 μg/ml DAPI (Beyotime). Images were collected and analyzed using a confocal microscope (Nikon A1R).

### Airway hyperresponsiveness

Airway hyperresponsiveness to methacholine challenge were measured after intranasal injection with 2 μg α-GalCer in 50 μl PBS for 24 h according to the published protocols (24). Briefly, 24 h after α-GalCer exposure, mice were anesthetized and surgically prepared with a tracheal cannula, then placed on a computer-controlled ventilator (UGO BASILE S. R. L, Italy). Measurements of airway pressure transducer, and airway resistance was monitored from pressure and volume data. Bronchospasm was induced with menthacholine in 0.9% NaCl at increasing concentration of 10, 25, and 100 mg/ml through a nebulization controller (emka) placed in line with the ventilator and delivered to the airway cannula for 25 s at a rate of 130 breaths/min. Airway resistance measurements were acquired at baseline and after each methacholine aerosol challenge for every 20 s in 5 min, ensuring that the parameters calculated were peaked. The resistance measurements were then averaged at each dose and graphed linearly (LR cmH_2_O/mL/s) along with the initial baseline measurement.

### BM chimera mice

Akt2^−/−^ mice were sublethally irradiated (6 Gy) and intravenously injected with a mixture 1 × 10^7^ total BM cells containing Akt2^−/−^ BM (expressing CD45.2) with wildtype BM (expressing CD45.1) at a 1:1 ratio. The recipient mice were analyzed 8 weeks later.

### Statistical analysis

Statistical significance was assessed by the two-tail student's *t*-test, or ANOVA was performed using Prism software (^*^p < 0.05; ^**^p < 0.01; ^***^p < 0.001).

## Results

### Akt2 deficiency reduces the accumulation of stage 2 iNKT cells

First, we examined the percentage and number of total iNKT cells in the thymus and spleen of Akt2 KO mice by using CD1d and TCRβ staining. Although the percentage was increased both in thymus and spleen (Figures 1A,B), the number of iNKT cells was decreased in thymus and spleen (Figure 1B). In order to determine the effect of Akt2 deficiency on the development of iNKT cells, we stained iNKT cells with the combination of CD1d and CD24 as well as CD44 and NK1.1 that defines the immature and mature iNKT cells including stage 0 to stage3 (Figures 1E,F). The percentage and number of stage 0, 1 and 3 of iNKT cells in Akt2 KO mice did not have difference either in thymus (Figures 1G,H,J) or spleen (Figures 1K,L,N). However, the percentage and number of stage2 iNKT cells were reduced significantly both in thymus (Figure 1I) and spleen (Figure 1M). RT-PCR was applied to confirm the *akt2* gene expression in iNKT and NKT17 cells that are concentrated in stage 2.We found that the *akt2* mRNA levels in iNKT cells were significantly higher than that of CD4^+^ T cells, which was close to that of NKT17 cells (Figure 1D). Because Akt2 KO mouse is a germline deletion, we made WT-WT and WT-Akt2 KO bone marrow CD45.1-CD45.2 mixed chimera mice, CD45.1 mice were used as the recipient mice to exclude the effect of environment. After 8 weeks reconstitution (Figure 1C), the mice were euthanized for flow cytometry analysis. We found that the percentage of CD45.2 Akt2 KO iNKT cells was increased and the number of that was decreased compared to that of CD45.2 WT iNKT cells (Figures 1A,B). Additionally only the percentage and number of CD45.2 stage 2 Akt2 KO iNKT cells were reduced (Figure 1Q). The percentage and number of CD45.2 stage 0, 1 and 3 of Akt2 KO iNKT cells was normal in the thymus (Figures 1O,P,R). All of these recapitulated the results from conventional Akt2 KO mice, which indicates the impact of Akt2 deficiency on iNKT development is cell autonomous. These results suggest that Akt2 controls the development and differentiation of stage2 iNKT cells.

**Figure 1:** Akt2 deficiency reduces the accumulation of stage 2 iNKT cells. **(A)** Flow cytometry of iNKT cells (CD1d-PBS57^+^TCRβ^+^) in the thymus (Thy) and spleen (Spl) from WT, KO, and chimera mice. **(B)** Percentages and absolute numbers of iNKT cells in the thymus and spleen from WT (*n* = 7), KO (*n* = 6), WT chimera mice (*n* = 4) and Akt2 KO chimera mice (*n* = 3). **(C)** CD45.1 and CD45.2 staining in thymus of chimera mice. **(D)** mRNA levels of *akt2* gene in CD4^+^T cells, CD19^+^B cells, iNKT cells, and NKT17 cells of WT mice. Expression of indicated mRNA from FACS-sorted CD4^+^T cells, CD19^+^B cells, iNKT cells and NKT17 cells of WT mice. **(E,F)** Thymic and splenic iNKT cell development stages. Percentages (**G–J**, upper panel) and absolute numbers (**G–J**, lower panel) of stages 0–3 iNKT cells from WT (*n* = 7) and KO mice (*n* = 7) in the thymus. Percentages (**K–N**, upper panel) and absolute numbers (**K–N**, lower panel) of stage 0–3 iNKT cells from WT (*n* = 6) and KO mice (*n* = 6) in the spleen. (**O–R**, upper panel) percentages and absolute numbers (**O–R**, lower panel) of stage 0–3 iNKT cells from WT chimera mice (*n* = 4) and Akt2 KO chimera mice (*n* = 3). *p < 0.05; **p < 0.01; ***p < 0.001 determined by the Student's *t*-test.

### Akt2 promotes NKT17 lineage differentiation

Previous research has shown that NKT cells can be categorized into NKT1, NKT2, and NKT17 lineages according to PLZF coupled with other signature transcriptional factor staining (6, 7). NKT1 cells are concentrated in stage 3, NKT17 cells are in stage 2, NKT2 cells are in stage 1, and stage 2 (6, 25). We investigated the effect of Akt2 deficiency on the differentiation of NKT1, NKT2, and NKT17 cells by PLZF staining together with T-bet, GATA3 and RORγt staining. Interestingly we found that the percentage and number of NKT17 (PLZF^+^RORgammat^+^) cells were significantly decreased in both thymus and spleen of Akt2 KO mice compared to that of WT mice (Figures 2A–C). Furthermore, the percentage and number of CD45.2 Akt2 KO NKT17 cells were also decreased compared to that of CD45.2 WT NKT17 cells in chimera mice (Figures 2A,B), which suggests that the effect of Akt2 deficiency on NKT17 differentiation is cell intrinsic. No difference was observed for the percentage and number of NKT1 cells either in thymus or spleen of WT and Akt2 KO mice (Figures 2A–C). Although the percentage of NKT2 cells was decreased in the thymus of Akt2 KO mice, the number of NKT2 cells was similar in WT and Akt2 KO mice (Figures 2A,B). We did not find any difference in the number and percentage of NKT2 cells in the spleen of Akt2 KO mice compared to that of WT mice (Figures 2A,C). Therefore Akt2 is indispensible for the generation of NKT17 cells.

**Figure 2:** Akt2 promotes NKT17 lineage differentiation. Cells were from WT and Akt2 KO mice. **(A)** Intracellular staining of PLZF, RORγt, T-bet, and GATA3 in iNKT cells from the thymus. Percentages and absolute numbers of NKT1, NKT2, NKT17 cells in the thymus (*n* = 6 mice per group) **(B)** and spleen (*n* = 4 mice per group) **(C)** from WT, KO, WT chimera mice (*n* = 3) and Akt2 KO chimera mice (*n* = 3). **(D–F)** Cytokine production by iNKT cells (gated on CD1d-PBS57^+^TCRβ^+^ cells) from the thymus (*n* = 5 mice per group) and spleen (*n* = 5 mice per group) after stimulation with PMA plus ionomycin for 5 h. **(G,H)** Cytokine production by iNKT cells from WT and Akt2 KO thymocytes stimulated with α-GalCer for 72 h and with PMA plus ionomycin in the last 5 h (*n* = 4 mice per group). **(I)** Critical role of Akt2 for PLZF localization to the nuclear bodies. MACS—enriched and FACS—sorted NKT17 cells from WT and Akt2 KO thymocytes(*n* = 3) were fixed and stained with a mouse anti-PLZF and Actin as primary antibody, detected with an Goat anti mouse secondary antibody. The nuclei were stained with DAPI. **(J)** Mean fluorescent intensity of cytoplasm and nucleus. *p < 0.05; **p < 0.01 determined by the Student's *t*-test.

The results above are in line with the reduction of stage 2 iNKT cells in Akt2 KO mice because NKT17 cells are concentrated in stage 2. To further investigate the effect of Akt2 deficiency on the production of cytokines in iNKT cells, we stimulated the iNKT cells with PMA and Ionomycin. We found that the production of TNFα, IFNγ, and IL-4 was similar in thymus (Figures 2D,E) and spleen (Figure 2F) of WT and Akt2 KO iNKT cells. However the generation of IL-17 was significantly decreased in Akt2 KO iNKT cells compared to that of WT iNKT cells both in thymus and spleen (Figures 2D–F). Because PMA and Ionomycin bypass the proximal signaling molecules and are not specific, we used a-GalCer as an agonist to stimulate iNKT cells and found that the IL-17 production was also significantly decreased in Akt2 KO mice (Figures 2G,H). These results correlated with the reduction of NKT17 cells in Akt2 KO mice (Figures 2A–C), suggesting that Akt2 is critical for the IL-17 production of iNKT cells. PLZF is a master transcription regulator of iNKT cell development (4, 5), and the nuclear localization of PLZF is important for iNKT-cell lineage development and effector function (26). We next examined the effect of Akt2 deficiency on the location of PLZF in the nucleus by confocal microscopy and PLZF staining. Interestingly we found that the staining of PLZF was distributed both in the cytoplasm and nucleus of WT NKT17 cells, but it was barely detectable in the nucleus of KO NKT17 cells (Figure 2I). The PLZF expression measured by mean fluorescence intensity (MFI) was comparable in the cytoplasm between WT and Akt2 KO NKT17 cells, but it was significantly lower in the nucleus of Akt2 KO iNKT cells (Figure 2J). These results suggest that the altered PLZF location in the nucleus of Akt2 KO iNKT cells may account for the abnormal central and peripheral development of iNKT cells.

### Loss of Akt2 reduces the proliferation and apoptosis of iNKT cells

Next we investigated the cellular mechanism for reduced absolute number of Akt2 KO iNKT cells by evaluating cell proliferation and apoptosis *in vitro*. First, we measured the proliferation of iNKT and NKT17 cells by examining the staining of Ki-67 and found that the percentages of Ki-67^+^ iNKT and NKT17 cells were decreased both in thymus and spleen of Akt2 KO mice (Figures 3A–F). Meanwhile we examined the apoptosis of total and stage 2 iNKT cells that take the majority of NKT17 cells by Annexin V and 7-AAD staining and found that the percentages of Annexin V or 7-AAD positive cells were decreased in total or stage 2 Akt2 KO iNKT cells of thymus and spleen (Figures 3G–O). The reduction of Annexin V positive cells in total and stage 2 iNKT cells was cell intrinsic (Figures 3J–L). Akt has been reported to inhibit FoxO-1 that trans-activates Bcl2 family proteins (27). To identify a pathway involved leading to reduced apoptosis in Akt2 KO iNKT cells, we examined the expression of the anti-apoptotic gene Bcl2 with intracellular staining. We found that the expression of Bcl2 was increased in both spleen and thymus Akt2 KO iNKT cells, which is cell intrinsic as well (Figures 3P–R). Therefore Akt2 deficiency diminishes the proliferation and apoptosis of Akt2 KO iNKT cells by promoting the expression of Bcl2.

**Figure 3:** Loss of Akt2 reduces the proliferation and apoptosis of iNKT cells. **(A)** Flow cytometry of Ki-67 cells gated on iNKT cells in the thymus. **(B,C)** Percentage of Ki-67 cells in the thymus and spleen (*n* = 3 mice per group). **(D)** Flow cytometry of Ki-67 cells gated on NKT17 cells in the thymus. **(E,F)** Percentage of Ki-67 cells gated on NKT17 cells in the thymus (*n* = 3 mice per group) and spleen (*n* = 3 mice per group). **(G)** Flow cytometry of Annexin V cells gated on the iNKT in the thymus. **(H,I)** Percentage of Annexin V cells in the thymus and spleen of WT (*n* = 3), KO (*n* = 3), WT chimera mice (*n* = 4) and Akt2 KO chimera mice (*n* = 3). **(J)** Flow cytometry of Annexin V cells gated on the stage2 (CD24^−^CD44^+^NK1.1^−^) iNKT cells in the thymus of WT, KO, and chimera mice. **(K,L)** Percentage of Annexin V cells of stage2 iNKT cells in the thymus and spleen of WT (*n* = 3), KO (*n* = 3), WT chimera mice (*n* = 4), and Akt2 KO chimera mice (*n* = 3). **(M)** Flow cytometry of CD1d cells gated on 7AAD cells in the thymus. **(N,O)** Percentage of CD1d cells in the thymus (*n* = 3 mice per group) and spleen (*n* = 3 mice per group). **(P)** Flow cytometry of Bcl2 cells gated on iNKT cells in the thymus. **(Q,R)** Overlaid histograms show expression of Bcl2.chimerachimera *p < 0.05; **p < 0.01, Student's *t*-test.

### Akt2 regulates the NKT17 differentiation by promoting the expression of ICOS

Previous research has shown that ICOS positively regulates the differentiation of NKT17 lineages (28). Signal transduction through ICOS results in the activation of PI3K (22), and a major pathway downstream of PI3K signaling is the Akt mediated inactivation of FoxO-1 (20, 29). Therefore, we investigated whether Akt2 has a feedback loop on the expression of ICOS in iNKT cells. Interestingly, we found that the percentage of ICOS positive iNKT cells was decreased in the thymus of Akt2 KO mice (Figures 4A,B) as well as the expression of ICOS (Figure 4C). The reduction of ICOS in the thymic Akt2 KO iNKT cells can be recapitulated in the spleen of Akt2 KO mice (Figures 4D–F). Additionally the reduction of ICOS positive iNKT cells and ICOS expression in thymus and spleen was repeated in CD45.2 Akt2 KO iNKT cells compared to that of WT iNKT cells in chimera mice (Figures 4G–L). c-Maf induced by ICOS regulates IL-21 production that, in turn, regulates the differentiation of T_H_17 cells (30), We examined the expression of c-Maf by intracellular staining and no difference was observed between WT and Akt2 KO iNKT cells (Figures 4M,N). We also examined other factors that may affect the differentiation of NKT17 cells, such as STAT3 and IL23R. STAT3 affects the expression of IL-17 by upregulating RORγt and RORα (31, 32). Although IL-23R is not required for the initial differentiation of NKT17 cells, it is essential for full and sustained differentiation of NKT17 cells (33). Therefore we examined the IL23R expression of iNKT cells and levels of pSTAT3 of thymocytes in Akt2 KO mice by using phospho flow after stimulation with PMA and Ionomycin. IL23R expression was not altered at all (Figures 4O,P), but we found that the levels of pSTAT3 were drastically reduced in Akt2 KO thymocytes (Figure 4T), which confirms the reduction of IL-17 signaling. We also used a-GalCer as an agonist to stimulate iNKT cells and found that the phosphorylation of STAT3 was also decreased by flow cytometry (Figure 4U). We also examined the mRNA levels of *icos, c-maf*, and *thpok* by real time-PCR. The mRNA levels of *icos* were significantly reduced in Akt2 KO iNKT cells (Figure 4Q), but no difference was observed for *c-maf* and *thpok* between WT and Akt2 KO iNKT cells (Figures 4R,S). To determine whether the reduction of NKT17 may affect iNKT cell function *in vivo*, we examined the airway hyperrepsonsiveness after induction with aerosolized methacholine. After 24 h α-GalCer challenge, both WT and Akt2 KO mice had significant elevations in their hyperresponsiveness to succeeding challenge does of methacholine compared to the baseline controls (Figure 4V). However, the hyperresponsiveness in Akt2 KO mice was significantly decreased compared with that of WT mice for the baseline although the increase was very similar in response to α-GalCer (Figure 4V). These results suggest that the deficiency of Akt2 affect the function of iNKT cells *in vivo*.

**Figure 4:** Akt2 regulates the NKT17 differentiation by promoting the expression of ICOS. **(A–F)** The percentages of ICOS of WT and Akt2 KO cells in thymus (*n* = 3 mice per group) and spleen (*n* = 3 mice per group) is shown. **(C,F)** Overlaid histograms show expression of ICOS in the thymus and spleen. **(G–L)** The percentages of ICOS of CD45.2^+^ cells in thymus and spleen of WT chimera mice (*n* = 4) and Akt2 KO chimera mice (*n* = 3) is shown. **(I,L)** Overlaid histograms show expression of ICOS in the thymus and spleen of chimeras. **(M,N)** The Flow cytometry of c-Maf and expression of c-Maf in the thymus. **(O,P)** Flow cytometry of IL-23R and expression of IL-23R in the thymus. **(Q–S)** mRNA levels of indicated molecules in WT and Akt2 KO iNKT cells. Expression of indicated mRNA from MACS- and FACS- sorted WT and Akt2 KO iNKT cells from freshly isolated thymocytes was quantified by real-time qPCR from three independent experiments. *p < 0.05; **p < 0.01, Student's *t*-test. **(T)** Flow cytometry analysis of the pSTAT3 for MFI in thymocytes from WT (*n* = 3) and Akt2 KO mice (*n* = 3). **(U)** Overlaid histograms show expression of pSTAT3 after α-GalCer stimulated 72 h. **(V)** Airway response to methacholine of WT (*n* = 3) and Akt2 KO mice (*n* = 3). LR, lung resistance from two independent experiments. *p < 0.05, Student's *t*-test.

### Akt2 couples with FoxO-1 to regulate the expression of ICOS in NKT cells

To further investigate the underlying mechanism of how Akt2 regulates the expression of ICOS via a feedback loop, we examined the expression of activated levels and location of FoxO-1 in iNKT cells by confocal microscopy and phospho flow. Akt has been reported to inhibit the downstream transcriptional factor FoxO-1 via the phosphorylation of FoxO-1 leading to exit from nucleus and degradation by ubiquitination in the cytoplasm (34). First, we examined the expression levels and location of total FoxO-1 in NKT cells by confocal microscopy after stimulation with α-GalCer. We found that the expression of total FoxO-1 was significantly higher in the nucleus of Akt2 KO iNKT cells compared to that of WT iNKT cells both in the non-stimulated and stimulated iNKT cells (Figures 5A–C). Furthermore, the levels of FoxO-1 in the nucleus of WT iNKT cells were significantly decreased after stimulation with a-GalCer compared to the non-stimulated WT iNKT cells, but no difference was observed for the FoxO-1 between non-stimulated and stimulated Akt2 KO iNKT cells. We also examined activated FoxO-1 after stimulation with PMA and Ionomycin by phospho flow. Not surprisingly we found that the levels of pFoxO-1 were significantly decreased in Akt2 KO iNKT cells (Figure 5D). ICOS is an upstream regulator of the PI3K-Akt axis and deficiency of ICOS may recapitulate the phenotype of Akt2 deficiency. We examined the activated levels and location of FoxO-1 in ICOS deficient iNKT cells with the same assay. Similarly to Akt2 KO iNKT cells, we found increased FoxO-1 in the nucleus of ICOS KO iNKT cells with or without stimulation compared to WT iNKT cells (Figures 5E–G). After stimulation, the decrease of FoxO-1 in the nucleus of WT iNKT cells can be seen but the levels of FoxO-1 stayed the same in ICOS KO iNKT cells (Figures 5E–G). Finally we found that the levels of pFoxO-1 were significantly reduced in ICOS KO iNKT cells by phospho flow after stimulation (Figure 5H). FoxO-1 has been shown to regulate the ICOS expression in Tfh cells, and therefore these results imply that Akt2 may couple FoxO-1 to regulate the ICOS expression in NKT cells.

**Figure 5:** Akt2 couples with FoxO-1 to regulate the expression of ICOS in NKT cells. **(A)** MACS—enriched and FACS—sorted iNKT cells from WT and Akt2 KO thymocytes were fixed and stained with a rabbit-anti-FoxO1 and AF488-Actin as primary antibody, detected with a goat anti rabbit secondary antibody. The nuclei were stained with DAPI. **(B)** MACS—enriched and FACS—sorted iNKT cells from WT and KO thymocytes were incubated with125 ng/mL α-GalCer for 3 d and then stained with FoxO1 and AF488-Actin as primary antibody, detected with a Goat anti mouse secondary antibody. **(C)** MFI of FoxO1 of iNKT cells in the thymus from the WT and Akt2 KO mice (*n* = 3) quantified with NIS-Elements AR 3.2 software. **(D)** Phospho flow analysis of the MFI of pFoxO-1(S256) in the WT and KO thymocytes. **(E)** MACS—enriched and FACS—sorted iNKT cells from WT and ICOS KO thymocytes were fixed and stained with a rabbit-anti-FoxO1 and AF488-Actin as primary antibody, detected with a goat anti rabbit secondary antibody. The nuclei were stained with DAPI. **(F)** MACS—–enriched and FACS—sorted iNKT cells from WT and ICOS KO thymocytes (*n* = 3 mice per group) were incubated with125 ng/mL α-GalCer for 3 d and then stained with FoxO1 and AF488-Actin as primary antibody, detected with a Goat anti mouse secondary antibody. **(G)** MFI of FoxO1 of iNKT cells in the thymus from the WT (*n* = 3) and ICOS KO mice (*n* = 3) quantified with NIS-Elements AR 3.2 software. **(H)** Phospho flow analysis of the MFI of pFoxO-1(S256) in the WT and ICOS KO thymocytes from three independent experiments. *p < 0.05; **p < 0.01, Student's *t*-test.

## Discussion

Cell metabolism has been implicated to have a critical role for the function of lymphocytes. mTORC is the central hub for the cell metabolism including mTORC1 and mTORC2 with the signature protein Raptor and Rictor. Akt is a key protein to connect mTORC1 and mTORC2. Akt is the downstream protein of Rictor after activation and further activates mTORC1. The role of Akt has been studied in T cells and B cells, but has never been investigated in iNKT cells. Our study reveals the role of Akt2 in the development and function of iNKT cells.

In our study we found that the deficiency of Akt2 causes the disruption of the homeostasis of iNKT cells. Although the percentage of total iNKT cells is increased, the total number of iNKT cells is reduced. This suggests that Akt2 deficiency affects conventional T cells as well and our results have shown that the percentage of CD4^+^ T cells is also reduced in the thymus of Akt2 KO mice (data not shown). Additionally the results from chimera mice have demonstrated that the increase of the frequency of iNKT cells in the thymus of Akt2 KO mice is cell intrinsic. Interestingly we found that the development of stage 2 iNKT cells was blocked, which leads to the reduction of NKT17 cells and IL-17 production correspondingly. It would be expected that if there are reduced iNKT17 cell numbers, there would be reduced IL17 production by total iNKT cells. Furthermore we analyzed the underlying cellular molecular mechanism of the reduction of total iNKT cells as well as NKT17 cells. Interestingly we found that both the proliferation and apoptosis is reduced in total Akt2 KO iNKT and NKT17 cells, which is cell autonomous. Surprisingly we found that Bcl-2 expression is higher in AKT2 KO iNKT cells, which is also cell intrinsic. But they would be more likely to survive than die since Bcl-2 is anti-apoptotic. This could be caused by the increased expression of apoptotic proteins in Akt2 KO iNKT cells, which is worthy to be pursued in the future research.

Furthermore we pursued the mechanism for reduced NKT17 cells in Akt2 deficiency and found that the reduction of ICOS generated by the negative feedback loop of Akt2 deficiency leads to the decrease of NKT17 generation. The increase of Akt2 has been shown to be correlated with the Th17-polarized WT T cells (35). It would be interesting to investigate the further underlying mechanism of how Akt2 regulates the expression of ICOS. However, there are a number of receptors that regulate the PI3K-AKT pathway, such as T cell receptor and IL7 receptor. While ICOS KO mice share a similar phenotype with AKT2 KO, currently we do not have direct evidence that ICOS-mediated AKT activation leads to these defects, it is possible that other receptors could be also involved.

FoxO-1 positively regulates the expression of growth factor receptors such as IL7R upon binding to the IL7 that inactivates FoxO-1 via a negative feedback loop (20). In our study, the deficiency of Akt2 led to reduced phosphorylation of FoxO-1 in iNKT cells, but the increased expression of FoxO-1 in the nucleus, which in turn led to a reduction of ICOS expression likely through a negative feedback loop. Therefore, we have revealed another negative feedback loop on the differentiation of NKT17 cells via the ICOS-FoxO-1 axis. ICOS signaling inactivates FoxO-1 via nuclear egress in naïve CD4^+^ T cells, which has been shown by the reduction of FoxO-1 in the nucleus after stimulation through CD3 and ICOS (20). The results of expression and location of FoxO-1 from ICOS KO mice have recapitulated that of Akt2 KO mice, which indicates that the ICOS-Akt2 axis regulates the expression and location of FoxO-1 in iNKT cells. FoxO-1 has been show to directly regulate the expression of ICOS via binding to the promoter of ICOS in Tfh cells (20). Therefore it would be interesting to confirm the binding of FoxO-1 to the promoter of ICOS in iNKT cells. Another interesting experiment would be to cross Akt2 KO mice with ICOS transgenic mice to examine if the defect of Akt2 deficiency could be rescued or not, such as the recovery of generation of NKT17 lineages and production of IL-17.

Another remaining question is the regulation of PLZF by Akt2. Our results have demonstrated that Akt2 regulates the expression and location of PLZF that is critical for the development of iNKT cells. Only few studies have mentioned the association between PLZF and Akt2. Akt has been reported to phosphorylate FoxO3a, which directly binds to the promoter of the PLZF gene (36). Akt might have direct or indirect modulation on PLZF by phosphorylation, which leads to the abnormal location of PLZF in the iNKT cells. Therefore it would be interesting to analyze the protein interactions between PLZF and Akt2 by using biochemical assays such as Co-Immunoprecipitation.

Overall our study links the metabolism molecules to the development and functions of iNKT cells and discloses the underlying molecular mechanism of distorted iNKT cell development in Akt2 KO mice. The deficiency of iNKT cells has been shown to lead to multiple diseases such as diabetes and cancer and our study suggests that it may be possible to design new therapeutic approaches to target metabolism pathways in clinical studies.

## Ethics statement

The project submitted by the research program and other information was reviewed and approved by the Ethics Committee of Chongqing Medical University. It is in line with the principles of medical ethics and the various requirements of Helsinki Declaration. The grade, quantity and specifications selected animal species were appropriate. The experiment meets the ethical standards of animal experimental research.

## Author contributions

CL carried out the initial analyses and drafted the initial manuscript. LN, XX, JW, LL, DY, and YJ performed the microscopic and flow cytometry assay. LW and CL conceptualized and designed the study, reviewed and revised the manuscript. All authors approved the final manuscript as submitted and agree to be accountable for all aspects of the work.

### Conflict of interest statement

The authors declare that the research was conducted in the absence of any commercial or financial relationships that could be construed as a potential conflict of interest.
